The article "Construction and Research of Constructive English Teaching Model Applying Multimodal Neural Network Algorithm" was published in 2022. Journal: Comput Intell Neurosci.

# Construction and Research of Constructive English Teaching Model Applying Multimodal Neural Network Algorithm

**DOI:** 10.1155/2022/9144656

**Published:** 2022-05-26

**Authors:** Nan Zhang, Hao Wang

**Affiliations:** ^1^Department of Foreign Languages, Jiujiang University, Jiujiang, Jiangxi 332005, China; ^2^Technical Service Center, Winner Technology Co., Inc., Shanghai 201210, China

## Abstract

This article draws on previous research on constructive English teaching models and uses multimodal neural network algorithm theory and constructive English teaching as the theoretical basis, experimental research method, questionnaire survey method, and evaluation method. In this article, we propose a multimodal neural network consisting of a multiscale FCN module and an LSTM module. The network focuses on both the multiscale geometric spatial features and the numerical time-dependent features of the time series curves, and with the comprehensive knowledge of their characteristics, it can better distinguish the classes to which the series belong. A large-scale perceptual field is achieved by null convolution in the model to ensure that the training pressure does not increase significantly. A series of experiments on the UCR dataset verifies the effectiveness and superiority of the model. Simulation experiments were conducted to build the proposed constructive English teaching model based on a multimodal neural network algorithm, and a test environment was built for use case testing. The experimental results showed that the algorithm can be better applied to constructive English teaching and has better adaptability and accuracy in various scenarios. At the end of the experiment, a posttest of grammar level was conducted in two classes to test whether the constructive English teaching model based on the multimodal neural network model could help students improve their English grammar skills. The results of the data analysis showed that the mean score of the experimental class was significantly higher than that of the control class, and the experimental class showed a more significant improvement, indicating that this new constructive English teaching model was beneficial to improving students' English grammar skills. The interaction strategy proposed under the constructive English teaching model can effectively improve the interaction between teachers and students. This positive feedback effect can provide front-line teachers with corresponding teaching references.

## 1. Introduction

Modern foreign language educators emphasize the whole process of language learning and strongly advocate that students should be exposed to and experience and understand the most realistic language situations in context and learn how to use the language fluently on that basis. The English program also strongly advocates the use of language teaching approaches and methods that emphasize the process of learning a language while enhancing students' learning outcomes, creating opportunities for students to communicate in authentic contexts as often as possible [1, 2]. Students are encouraged to discover language rules and gradually acquire language knowledge and skills through active inquiry and cooperation under the guidance of the teacher and to develop an effective self-inquiry learning strategy through continuous emotional and attitudinal adjustment, thus developing their independent learning skills. In this case, teachers should pay attention to the cognitive level of junior high school students and their physiological and physical characteristics, design a variety of learning methods, motivate students to learn, and train students to learn English practically through a variety of ways. Teachers use questions to create situations, introduce students to the imagination about the future created in the previous lesson, activate students' attention, and let them think about the problems at the introduction stage of the class, enter the learning state with the problems, avoid the traditional classroom single-issue lecture, and let students be fully prepared for the psychological learning [3]. It allows students to gain a sense of accomplishment and boost their self-confidence while exploring on their own. The deep learning method is fault-tolerant to the input and can take the unaligned complete time series as input. It can automatically extract features from the input data and explore the key features of the original data at various scales without missing detailed information [4]. Therefore, among the two, the deep learning model performs relatively well, and in terms of a single model, the classification correctness of the deep learning model exceeds that of most feature representation-based methods. In addition, there are also some methods based on the above two approaches, and by fusing multiple feature representations or multiple types of methods, a model capable of learning time series feature information from multiple perspectives simultaneously is obtained [5].

The article "Construction and Research of Constructive English Teaching Model Applying Multimodal Neural Network Algorithm" was published in 2022. Journal: Comput Intell Neurosci.

The scientific and reasonable design of teaching activities and the arrangement of teaching programs are the basis for the realization of the teaching effect of innovative teaching methods. In the innovative teaching method, teachers have to realize the multirole transformation of designer, guide, observer, and consultant [6, 7]. The requirements of analyzing and understanding teaching purposes, arranging teaching contents reasonably, changing teaching activities flexibly, demonstrating and explaining the rules of activities, and observing teaching feedback in time pose higher challenges to teachers' professional quality level. Teachers should not only keep learning pedagogy, psychology, and other professional knowledge but also keep improving their ability of language expression, analysis, and observation to meet the requirements of innovative teaching methods. Moreover, the improvement of teachers' professionalism will promote the effective improvement of teaching levels beneficial to the integration of games and teaching and presenting them in the classroom [8]. With the increasing degree of information technology today, China also has a lot of teaching video websites that can provide quality courses with rich and diverse teaching resources, all of which can provide a resource base for the development of the flipped classroom teaching model. Thanks to the support of these network platforms. This article focuses on constructing a constructive English teaching model with a multimodal neural network algorithm for teaching practice [9]. It helps to help domestic teachers better understand the content of innovative teaching methods, explore the application form of innovative teaching methods, help educational scholars better explore the concept of constructive English innovative teaching, and play a role in promoting the application of constructive English innovative teaching methods [10].

English is a part of students' learning, and the so-called laying a good foundation is the key. This study combines multimodal neural network algorithms with traditional constructive English teaching to remedy the shortcomings of the traditional classroom teaching process, such as insufficient teaching dynamics and lack of student motivation, to improve the efficiency of English teachers' teaching and students' learning. This thesis is divided into five parts [11]. The first part is the introduction, which firstly introduces the research background of this dissertation, secondly introduces the research purpose of this dissertation, next elaborates the research significance of this dissertation from two aspects, and finally introduces the framework of this dissertation: theoretical significance and practical significance. The second part is the related research section, multimodal feature fusion, which details the basic methods for conducting feature fusion and using features to fuse constructive ELT features to form multimodal features. Then the current status of research on constructive ELT models at home and abroad is presented and evaluated. The third part of the article is a study on constructing a constructive ELT model based on a multimodal neural network algorithm, multimodal feature fusion, detailing the basic methods of conducting feature fusion, using feature fusion image features to form multimodal features, and studying the evaluation of constructive ELT models. The fourth part is the result analysis section, which verifies its effectiveness and superiority by implementing various experiments and comparisons on the UCR time series dataset. Experimental validation of the model was conducted on the UCR dataset, and an attempt was made to use the model for aeroengine air circuit troubleshooting problems, with good results in both sets of experiments. Finally, the mechanism of the model's functioning is analyzed using the intermediate process data of the two experiments. The fifth part summarizes and analyzes the construction of a constructive English teaching model with a multimodal neural network algorithm and the outlook.

The article "Construction and Research of Constructive English Teaching Model Applying Multimodal Neural Network Algorithm" was published in 2022. Journal: Comput Intell Neurosci.

## 2. Related Research

One of the common approaches to overcome the shortcomings of time series data is to transform the original sequence into a feature space where differences can be more easily detected for representation. In this space, the feature representation of the time series may be discrete, of lower dimensionality, or without alignment problems so that more conventional classifiers can be used to solve the time series classification problem [12]. There are a large number of methods for classification based on feature information of time series, which construct a variety of feature representations. Since the RNN family of networks is designed for prediction problems and is difficult to train with the risk of gradient disappearance and gradient explosion, there are actually few methods that use networks such as LSTM alone as time series classifiers [13]. LSTM and GRU are generally used as temporal feature extractors or in combination with other deep learning models. Wang et al. directly used the integration over time of each neuron output in the ESN storage pool and the sum of all neuron outputs in the same moment state as input to the decision layer to give classification results [14]. Xu et al. used the ESN as a temporal feature extractor, constructing the ESN output as a two-dimensional matrix [15]. Zhang et al. used ESN as a temporal feature extractor and constructed the output of ESN as a two-dimensional matrix, followed by CNN for secondary feature extraction and classification [16]. Teachers can base their instructional design on these four basic elements and design more relevant and effective motivational strategies based on students' motivational profiles and the characteristics of the required content, when appropriate. The four elements represent the four main types of motivation strategies, and only a flexible and appropriate instructional design based on the four basic elements can effectively motivate students to learn and optimize teaching efficiency [17].

The article "Construction and Research of Constructive English Teaching Model Applying Multimodal Neural Network Algorithm" was published in 2022. Journal: Comput Intell Neurosci.

The learning environment is very important for English learning, and schools should provide a relative environment for students to learn English better, carry out more extracurricular activities about English, and encourage students to learn English knowledge by participating in activities so that students' initiative to learn English can be improved and thus better implement constructive English teaching [18]. Li et al. argued that the essence of teacher-student interaction is a concept of teaching and learning. In the process of teaching, it is not only the teacher who transmits knowledge to students, but also the teacher and students learn from each other, enrich themselves, and achieve mutual benefits of teaching and learning and the common development of teachers and students, which is the interaction and influence between teachers and learners [19]. Li et al. added a multiscale conditional random field (CRF) to the network structure to optimize the details of the prediction results by one [20]. Jeon et al. were inspired by the traditional structure from motion approach and proposed a new idea to achieve unsupervised training of deep prediction networks [21]. With the powerful modeling ability of deep neural networks, these single-view depth prediction methods based on deep learning can obtain dense and smooth prediction results [22, 23]. The deep learning technology itself is a data-driven recognition process. By adding image data samples with corresponding feature skew, change, and noise, the model can better identify these biological features in nonstandard states to better improve user experience [24].

The research on innovative teaching methods by educators is constantly progressing and developing, and various types of innovative teaching methods are constantly being innovated according to different contemporary contexts and teaching environments [25]. However, the focus has always been on student-centered teaching methods that are suitable for the current physical and mental characteristics of students based on cognitive theory. Various aspects such as teaching environment, the content of teaching materials, teaching objectives, classroom interaction, teacher quality, and student characteristics have been studied and discussed. However, the multimodal neural network algorithm innovative teaching method is the first time that a systematic multidimensional and multifaceted analysis of various elements in teaching has been conducted in multiple regions, and the relevant theoretical framework has been summarized and sorted out [26, 27]. It lays a theoretical foundation for innovative teaching methods and facilitates the understanding and application of innovative teaching methods by education scholars. The multimodal neural network algorithm considers RGB, depth, and optical flow data streams simultaneously and proposes the following four improvement strategies without changing the core structure of the neural network: first, a layering strategy is proposed to divide the video into several subsequences, with each subsequence as a complete input unit, which facilitates the model to capture more local information of the video. Second, the input to the model is normalized by combining the optical flow-based uniform random sampling method with the multimodal network in a hierarchical structure of input modules [28, 29]. Engaging introductions maximize student interest and engage students in classroom teacher-student interactions. The exact goal provides the ultimate purpose of interaction between teachers and students [30]. Appropriate pretests can allow teachers to understand the actual situation of students and also allow students to review what they have learned. Participatory learning allows students to interact with teachers and students as much as possible and learn easily through interaction. A timely posttest can facilitate teachers' teaching evaluation and reflection.

The article "Construction and Research of Constructive English Teaching Model Applying Multimodal Neural Network Algorithm" was published in 2022. Journal: Comput Intell Neurosci.

## 3. Research on Constructing a Constructive English Teaching Model Based on a Multimodal Neural Network Algorithm

### 3.1. Features of Constructive English Teaching

In actual teaching, teachers cannot use only one pedagogy to teach. Pedagogies are not separate from each other. They are influenced by each other, a combination of mutual feedback, and their continuous unity constitutes the combination, which leads to the formation of pedagogical orientations. In a broader sense, pedagogical orientation is also included in the combination of pedagogies so that the long-term educational goals can be met. The emphasis on the combination of pedagogies is because different pedagogical orientations lead to different teaching and learning processes. These three combinations specifically refer to the combination of pedagogical tools, pedagogical methods, and pedagogical content, all of which are extremely helpful in improving the quality and enriching the content of teaching and learning. Professional teachers and teaching strategies are the basis for identifying the design and implementation of pedagogy. The identification of pedagogy is a prerequisite for the design of classroom activities. Teachers should understand the principles and conditions of identifying pedagogy when designing classroom activities.

The article "Construction and Research of Constructive English Teaching Model Applying Multimodal Neural Network Algorithm" was published in 2022. Journal: Comput Intell Neurosci.

The key to the school context is in the school and the educational system; for example, the organizational culture, practices, and collective behaviors of the school are all important causes of impact. Lauri has pointed out that the obstacles to effective teaching and learning are not only in the classroom but also in the organizational environment, which may also hinder the outcome of teaching and learning, so teachers need to take a comprehensive look at the possible influences on student learning as much as possible. Student background refers to the fact that there are differences in the social or cultural backgrounds of individual students and that students from relatively poor backgrounds need relatively more support so that innovative teaching methods cannot only use inquiry or discovery methods, which may not apply to all students. In the teaching application, change is reflected in the change of roles; students and teachers exist in equally important roles; in teaching activities, students are also participants, teachers should focus on the feedback given by students in teaching activities; the change of teachers is also reflected in the teaching application of teaching, from existing theories, resources, and models and individual teachers should obtain information from them to develop teaching concepts. Teachers should use the constructive English teaching framework to design the overall structure of teaching activities and then use innovative teaching methods to achieve teaching goals and enrich the whole teaching process. The constructive English teaching model is shown in Figure 1.

Knowledge originates from and is rooted in real activities and situations. The theory emphasizes that knowledge is attached to activity situations and the creation of situations should be based on learners' life backgrounds and existing experiences and students' experience and practice in the situations to complete the construction of knowledge. Knowing and doing are interactive: students learn in contextual activities, combine their own experiences, and acquire knowledge, which is dynamically generated in context; i.e., knowledge is contextualized and learning is based on context. Meaningful negotiation: teachers create and design different learning contexts in class to meet the needs of students at different levels, which helps students of different levels and personalities to interact actively and learn cooperatively. Students know what to do by actively participating in hands-on activities, sharing common insights, and having common learning goals in reasonable contexts created by the teacher. In contextualized instruction, students are real participants in the classroom, not observers, and they cannot be involved in all but only some of the activities. Teachers should create learner-centered contexts with similarities to learners' daily life scenarios and encourage and guide learners to engage in inquiry-based and creative learning in actual activities, with mutual interaction and active interaction between teachers and students.

The article "Construction and Research of Constructive English Teaching Model Applying Multimodal Neural Network Algorithm" was published in 2022. Journal: Comput Intell Neurosci.

For continuous data such as time series, ELTs, and various types of signals, the use of null convolution for their perception approximates the mathematical use of equally spaced interpolation to approximate the shape of a function curve, and the information from a few interpolation points can be used to obtain rough characteristics of the data. As shown in Figure 2, taking the GunPoint dataset as an example, the left-hand side gives the data distribution of the two categories of instances on the most distinctive subsegments; the upper and lower plots on the right-hand side show the perceived data at a void rate of *d* = 4 and *d* = 6, respectively, and it can be seen that the points learned by jumping to the ground still roughly reflect the distribution characteristics possessed by the complete data. First, set the general structure of the model, keep this part of the structural hyperparameters unchanged for all data sets, then perform a restricted grid search for some hyperparameters for each dataset, and perform a restricted grid search for some the hyperparameters for each dataset. Performance evaluates it, keeping the hyperparameter combination that gives the best overall performance.

### 3.2. Constructing a Constructive English Teaching Model with a Multimodal Neural Network Algorithm

To strengthen the network's ability to apply this kind of picking distribution, during training, we randomly select a threshold value based on the gradient of the RGB image and randomly sample the depth labeled data to obtain the sparse depth as shown in equation (1), where EI(*m*) denotes the grayscale image corresponding to the input RGB image with the modal pan of the gradient at position *m*, which is a uniform random machine variable:

(1) $$\begin{array}{c} G\left(m\right)=\left\{\begin{array}{cc} 0, & |\text{EI}\left(m\right)|\leq \varphi ,\\ 1, & |\text{EI}\left(m\right)|>\varphi . \end{array}\right. \end{array}$$

For each node to be computed, the node pair with the smallest distance from it is selected in the window to form a relatively aligned node pair, and the minimum distance value is used as the local distance between the node pairs. Using dynamic planning and recursive operations, the node pairs that should be aligned can be continuously determined to shorten the size of the sequence to be processed. The final GHW distance is the accumulation of the local distances of all aligned node pairs, which is calculated as shown in equation (2). The flexible matching of node pairs and the reusability of nodes enable the GHW algorithm to adapt to the distance calculation between unaligned and unequal sequences to a certain extent, making it the most commonly used direct distance measure. The gis denotes the distance between the current corresponding node pairs.

(2) $$\begin{array}{c} \text{GHW}\left(M_{X}^{2},N_{Y}^{2}\right)=\text{gis}\left(m_{X},n_{Y}\right)+\left\{\begin{array}{c} \text{GHW}\left(M_{X-1}^{2},N_{Y-1}^{2}\right),\\ \text{GHW}\left(M_{X}^{2},N_{Y-1}^{2}\right),\\ \text{GHW}\left(M_{X-1}^{2},N_{Y}^{2}\right). \end{array}\right. \end{array}$$

The size of the perceptual field of the null convolution is based on the first metric, which can be calculated according to equation (3). *N* is the size of the defined convolution kernel; *P* is the expansion rate; *N*^″^ is the size of the conventional convolution equivalent to this null convolution. Using atrous convolution to extract features from one-dimensional continuous data in a large span is an effective method, and it is applied to time series data to extract long-term features within a large period. The way to jointly control the receptive field by adjusting the size of the convolution kernel and the dilation rate also inspires the structural design of the multimodal model.

(3) $$\begin{array}{c} N^{\prime \prime }=N+\left(N-1\right)*\left(P-1\right). \end{array}$$

The network structure of both FCN and LSTM-FCN models is kept constant for all datasets, and then for each dataset, a restricted grid search is performed for some of the hyperparameters, and it is evaluated based on its overall performance on all datasets, and the combination of hyperparameters that makes the best overall performance is retained. The network structure of both FCN and LSTM-FCN models when they are close to the best state and the hyperparameters are detailed in Table 1.

The article "Construction and Research of Constructive English Teaching Model Applying Multimodal Neural Network Algorithm" was published in 2022. Journal: Comput Intell Neurosci.

In this article, we choose to fuse the output data of FS8, the third fully connected layer in the multimodal model, where the output of the FS8 layer is FS(HI, *ψ*)=∑_*i*=1_^4^*h*(CS(*X*_*i*_, *ψ*) and *ψ* denotes the set of network parameters for the current iteration of the multimodal model. Since all sequences belong to the same video, the class to which the sequences belong should also be the same. Therefore, the elements can be merged and the output of the sequence fusion part, as in the following equation:

(4) $$\begin{array}{c} \text{HP}=\sum_{i=1}^{4}h\left(\text{CS}\left(X_{i},\psi \right)\right.. \end{array}$$

Given the input data *X*, a multimodal neural network classification model will estimate the probability *F*(*Y*=*K|X*) that data *x* belongs to each category *K*. That is, suppose a function for the input *x* will output a k-dimensional vector to represent the probability that *x* belongs to each type, assuming that the function *h* (*x*) takes the form shown in the following equations, where *ψ*={*ψ*_*i*_},  *i*⊆[1, *k*] model parameters and *Y* denotes transpose:

(5) $$\begin{array}{c} M\left(\psi ,X^{k}\right)=\left[\begin{array}{c} F\left(Y^{k}\right)=11*X^{k};\psi \\ F\left(Y^{k}\right)=22*X^{k};\psi \\ F\left(Y^{k}\right)=kk*X^{k};\psi \end{array}\right]=\frac{M\left(\psi +1,X^{k+1}\right)}{\sum_{i=1}^{K}\psi^{k,X^{i}}}. \end{array}$$

Due to a large amount of data in practical applications, there are some special cases after the kernel function transformation still cannot find a suitable hyperplane to perfectly distinguish the two classes of data, so the SVM allows a small portion of samples to be in the region of another class through the relaxation variables as a cost to penalize the objective function, thus limiting the SVM model to include too many of these special cases. The objective function is changed to, as in the following equation, where *Q* is the penalty factor, which needs to be set artificially and *ω*(*i*, *m*, *n*) is the variable to be optimized:

(6) $$\begin{array}{c} F\left(\psi \right)=Q*\sum_{i=1}^{N}\omega \left(i,m,n\right)*P\left(i,\psi^{Y},\beta \right)+\frac{\text{max}{\left\|\psi \right\|}^{2}}{2}. \end{array}$$

The adversarial loss function is mainly responsible for reconstructing the scene details using adversarial training. *G*(*d*) is a G1 reconstruction loss function that directly supervises the network training to minimize the error between the mesh output and the labeling. It represents the classic multimodal neural network TSC model, in which the input information of MCNN contains the representation of time series under various downsampling rates, which is equivalent to multiscale spatial feature learning. The multiscale convolutional FCN model with different algorithm structures in this article is not enhanced by the LSTM module.

(7) $$\begin{array}{c} G\left(d\right)=∐\left(m,n\right)*\left\|n-H\left(m\right)\right\|. \end{array}$$

The adaptive smoothing loss function *G*(*s*) imposes an adaptive penalty on the magnitude of the gradient *δ*_*k*_*∗M*^*X*−1^ of the network output, as shown in the following equation, where *δ*_*k*_*∗N*^*Y*−1^ represents the gradient of the depth initialization result:

(8) $$\begin{array}{c} G\left(s\right)=∐\left(M^{X},N^{Y}\right)*\left\|\delta_{k}*M^{X-1}*\tau^{-\delta_{k}*N^{Y-1}}\right\|. \end{array}$$

In the second stage, the CNN and BPNN are trained to a better state using the training set, and their scores for determining the likelihood of the validation set and test set samples belonging to each category are obtained; after that, the body of evidence of D-S evidence theory is constructed from this score as the information source. In the process, the integration of the model to the validation set can be used to adjust the two information sources to make the model better integrate the test set; finally, the multimodal information in the form of evidence body is integrated according to the synthesis rules to form a new basic probability distribution, and the final discriminant results are generated according to the decision rules. The overall flow of the algorithm is shown in Figure 3.

The article "Construction and Research of Constructive English Teaching Model Applying Multimodal Neural Network Algorithm" was published in 2022. Journal: Comput Intell Neurosci.

### 3.3. Evaluation of the Constructive English Teaching Model

The outcome evaluation metrics include the overall correct or error rate of classification, the number of best results achieved, the average ranking of the results, and the average category error rate MPEC. MPEC can be used to expect the classification error rate of the model for a single category, which is defined in the following equation, where *n* denotes the number of datasets, *i* is the *i*th dataset, *i*⊆[1, *N*], *N*(*e*)_*i*_ denotes the error rate of the *i*th dataset; *N*(*e*)_*i*_ denotes the number of categories in the *i*th dataset, and RPQ denotes the error rate equally spread over each category:

(9) $$\begin{array}{c} \left\{\begin{array}{c} {\text{RPQ}}_{i}=\frac{N{\left(e\right)}_{i}}{N{\left(c\right)}_{i}}\\ {\text{MRPQ}}_{i}=\frac{\sum_{i=1}^{N}\text{RPQ}}{N} \end{array},\;\right.i\subseteq \left[1,N\right]. \end{array}$$

The Friedman rank-sum test based on the algorithmic ranking is used to evaluate overall whether there are differences in the performance of multiple models on multiple datasets. The rank ranks the classification accuracy of a particular dataset among all models involved in the comparison, so the rank-sum can be calculated using the average rank and the total number of datasets that have been derived. Assuming that *k* algorithms are compared on N datasets, the statistic *G*(*k*) constructed in the Friedman test is calculated as shown in the following equation, where *ψ*(*G*)_*i*_ is the average rank of the *i*th algorithm on all datasets:

(10) $$\begin{array}{c} G\left(k\right)=\frac{\left(N-1\right)\psi {\left(G\right)}^{2}}{N\left(k-1\right)-\sum_{i=1}^{N}\psi {\left(G\right)}^{2}}. \end{array}$$

The evaluation scale is designed based on the four elements of the multimodal neural network model, and all four basic elements are presented in the evaluation scale. The scale is designed mainly to enable teachers to summarize and reflect on the defects and shortcomings of the activities through students' evaluation of the teachers' teaching design, i.e., the degree of classroom pacing, to further improve the teaching design, optimize the implementation process of the activities, and provide a timely and effective basis for improving the vitality and efficiency of classroom teaching more effectively. The details are shown in Table 2. Teachers and group members observe each other. Each member of the group conducts self-evaluation and mutual evaluation on the mastery of vocabulary and grammar in the course, the degree of contribution and participation in group activities, and the ability to express and communicate in situational dialogue performances. Teacher evaluation: the author chooses the form of evaluation scale to conduct the summative evaluation of this lesson. In the selected evaluation scale, the evaluation is divided into multiple subjects and nine aspects, including self-evaluation, other evaluation, and teacher evaluation. This makes the evaluation more comprehensive, more authentic, and effective. In the teacher evaluation part, teachers should encourage and affirm students to enhance their learning satisfaction.

The article "Construction and Research of Constructive English Teaching Model Applying Multimodal Neural Network Algorithm" was published in 2022. Journal: Comput Intell Neurosci.

The summative evaluation is applied to the evaluation of the teaching phase or after the achievement of the objectives of the whole course. It is a comprehensive and integrated evaluation and recommendation for each student subject from the perspective of each dimension and each participant in the teaching activity. This makes the evaluation multifaceted and multielement, which improves the traditional teacher's subjective evaluation system, prevents students from being prejudiced in teaching activities, and greatly improves the teaching evaluation system. Each student's performance in teaching activities is seen by the teacher and other members, and in the communication and collaboration, each student can express their ideas and opinions equally and freely and is no longer prevented or judged unilaterally. While communicating in groups, they can build on their strengths and quickly come up with ideas or solutions to problems. All these promote the balanced development of fairness and efficiency and increase the understanding and affirmation among students and between teachers and students.

## 4. Analysis of Results

### 4.1. Analysis of Multimodal Neural Network Algorithms

In this article, two multimodal English feature evaluation structures based on 5-layer convolutional neural networks are designed. Two fusion methods are used in the fusion approach: the first fusion method is to add the corresponding elements of each feature map (G1 for short); the second method is to connect each feature map directly (G2 for short). The experimental results of the two multimodal English feature structures with different fusion methods are shown in Figure 4. As can be seen from Figure 4, the overall evaluation effect of Structure II is slightly higher than that of Structure I. The average evaluation rate of StructureI-G1 is 98.39% and that of Structure I-G2 is 97.87%. The average evaluation rate of Structure II-G1 is 98.26% and that of Structure II-G2 is 98.25%. But the evaluation results of either multimodal English feature structure are higher than the evaluation results of unimodal 97.89%; i.e., the accuracy of multimodal evaluation methods is better than that of unimodal evaluation methods.

The article "Construction and Research of Constructive English Teaching Model Applying Multimodal Neural Network Algorithm" was published in 2022. Journal: Comput Intell Neurosci.

To study the effect of the feature fusion method of primary features in the convolutional neural network on the performance of multimodal evaluation, based on the evaluation structure of Structure II, this article proposes a dual feature fusion mechanism, in which the first layer of convolution is followed by the first fusion of three modal data or any two of them, and there are four fusion methods in the first fusion, which are referred to as Structure II-M1, Structure II-M2, Structure II-M3, and Structure II-M4 in the following experiments. Based on the above four double feature fusion methods, this article uses the multimodal fusion method to compare the four fusion methods, and the experimental results are shown in Figure 5. The evaluation results of these four fusion methods are relatively stable, all of them above 93.58%. Among them, the evaluation effect of Structure II-M4 is the most outstanding, so we can infer that the richer the fusion features at the first primary feature fusion, the better the multimodal evaluation performance. In the multimodal evaluation method, the dual feature fusion method can improve the multimodal evaluation performance, and the richer the primary feature fusion, the higher the multimodal evaluation accuracy. In summary, the multimodal constructive English teaching method based on the convolutional neural network proposed in this article can get a high evaluation rate and can effectively accomplish the unimodal or multimodal constructive English teaching tasks.

### 4.2. Simulation Analysis of Constructive English Teaching Model

As shown in Figure 6(a), the difference between the English scores of the two classes is 1.5124. As shown in Figure 6(b), the mean score and standard deviation of the experimental class are higher than those of the control class, which indicates that the test scores of the experimental group are unevenly distributed. The reason for this situation is that some students could not adapt to the innovative teaching method, but overall, the test scores of the experimental group improved.

The article "Construction and Research of Constructive English Teaching Model Applying Multimodal Neural Network Algorithm" was published in 2022. Journal: Comput Intell Neurosci.

In Figure 7, we found that after the chi-square test, *F* = 0.6892, the value of the chi-square test result Sig = 0.7145 is greater than 0.06, and we believe that the overall variance of the English scores of the two experimental subjects is equal. After that, the *t*-test was executed to find *T* = 0.143, and since Sig = 0.6751 is less than 0.08, it is evident that there is some variability between the experimental class and the control table scores. Based on the analysis of the experimental data, we can conclude that the innovative teaching method has an improving effect on the English performance of the students in the experimental class. Because of the uneven distribution of English scores in the experimental class, it can be presumed that some students did not adapt to and approve of the innovative teaching method.

Both classes belonged to the same level before the experiment, and their language expression levels were the same. In the process of experimenting, English teaching in both classes was the same except for the differences in teaching methods, and through the semester-long experimental activities, both were improving in terms of their overall English proficiency, although the experimental class using the innovative teaching method had a significant improvement compared to the control class. Therefore, it was possible to obtain results that the use of the innovative teaching method in the English classroom process was effective in improving the achievement scores of the students compared to the previous teaching method.

### 4.3. Evaluation Analysis of Constructive English Teaching Model

In the course of the experiment, the teacher-student interaction strategy proposed by the constructive English teaching model was used in the experimental class, while the ordinary teaching method was used in the control class. During the experiment, the author recorded the teacher-student interaction behavior of the experimental class not only through classroom observation but also by using the tool Flanders analysis matrix. The results of the experiment for the control class and the experimental class are shown in Figure 8. The difference between the students in experimental class and control class was 0.21, indicating that the teacher was consistently receptive to the students' perspectives. The difference between the experimental class and the control class was 2.25, indicating that the teacher in the experimental class asked students more questions or the teacher asked students for a longer duration, creating more opportunities for student-teacher interaction. The difference of 6 between the students in Experimental Class and Control Class indicates that the English teacher in experimental class spent less time lecturing by herself and more time interacting and discussing with students, and the classroom was student-oriented; hence, the behavior of teacher-student interaction increased. The difference between students in the experimental class and control class is 0.002, which indicates that the teacher's instructions are emotionally stable. The difference of 0.12 between the students of the experimental class and control class indicates that both experimental classes had little time for teacher criticism and the teacher gave more encouragement to the students. After the experimental class adopted the strategies of teacher-student communication in the middle school English classroom proposed under the constructive ELT teaching model, the teacher-student interaction atmosphere was good, the teacher praised students' behavior more, students' self-efficacy was high, the teacher-student interaction lasted longer, and students actively participated in the interaction.

The article "Construction and Research of Constructive English Teaching Model Applying Multimodal Neural Network Algorithm" was published in 2022. Journal: Comput Intell Neurosci.

As shown in Figure 9, it can be observed that the multimodal neural network-based algorithm outperforms the other five methods, among which FLiXT II, AMRL II, and XDETVP II are the methods proposed by the top three teams that won the challenge, respectively, while the algorithm in this article adds the above four improvement strategies to the original multimodal model. The evaluation rate obtained by this algorithm on the IsoGD III validation set is 2.1 percentage points higher than the 54.2% obtained by the first-place team, which proves that the algorithm in this article has a good research prospect and affirms the research work we have done.

For the analysis of the experimental results, the constructive ELT evaluation algorithm designed in this article is based on a multimodal neural network, in which the constructive ELT actions have a good evaluation effect and meet the basic needs of everyone. Moreover, when analyzed in terms of evaluation rate, we found that if the constructive ELT actions have simple strokes, they seem to have a higher evaluation rate than the general Arabic numeral constructive ELT activities. Therefore, this means that if the constructive ELT actions have simpler strokes in expression, then there will be a higher success rate through constructive ELT evaluation; if the constructive ELT actions have very complex and cumbersome strokes, it may not be easy to achieve success using constructive ELT evaluation, which will easily lead to wrong results. Analyzing the relevant evaluation results, it is found that the algorithm designed in this article, which is based on the multimodal neural network using a constructive ELT evaluation algorithm, has a more accurate evaluation rate, and the evaluation methods of FLiXT II, AMRL II, XDETVP II, and constructive ELT evaluation algorithm based on multimodal neural network is not difficult to implement, and it will have certain self-organization and self-learning level. This shows that the multimodal neural network-based constructive English teaching evaluation algorithm designed in this article is feasible for constructive English teaching evaluation.

The article "Construction and Research of Constructive English Teaching Model Applying Multimodal Neural Network Algorithm" was published in 2022. Journal: Comput Intell Neurosci.

## 5. Conclusion

In this article, two new TSC methods are proposed, starting from the aspects of learning data features comprehensively and making each deep network fully functional. Along the lines of this article, there are still some issues worth further research in the future: for the first method, the exploration of more scales and how to generate multiscale perceptual fields from the combination of traditional convolution and null convolution can be carried out, and the joint learning of more types of features, such as adding BPNN structure to learn the overall distribution of sequence features, can also be attempted; for the second method, the fusion of other simple structure and good performance can be considered. For the second approach, decision-level fusion can be considered for other deep networks with simple structures and good performance, and other methods other than evidence theory can be used for information fusion. The teaching activities of innovative teaching methods are rich and diverse, and students have the opportunity to show their various strengths and get the satisfaction of knowledge displayed from the activities, which helps students to improve their learning confidence, motivate their learning, and develop good learning quality. Innovative teaching methods in teaching practice more often use games, competitions, and other teaching activities; these group-based teaching activities can make students' listening, speaking, reading, and writing skills get balanced exercise, and interactive activities can give teachers and students more opportunities to communicate and cooperate, improve English core literacy, and promote the effective improvement of students' comprehensive ability. Teachers should not only keep learning pedagogy, psychology, and other professional knowledge but also keep improving their ability of language expression, analysis, and observation to meet the requirements of innovative teaching methods. Moreover, the improvement of teachers' professionalism will promote the effective improvement of teaching levels. The performance in network structure, training time, and decoding time has been greatly improved because real time is a major fundamental for constructive English teaching to reach its peak, and the reduction of training decoding time can make the constructive English teaching model more intelligent. Therefore, using more advanced neural network models can be the next research direction.

The article "Construction and Research of Constructive English Teaching Model Applying Multimodal Neural Network Algorithm" was published in 2022. Journal: Comput Intell Neurosci.

## Figures and Tables

**Figure 1:** Constructive English teaching framework.

**Figure 2:** Extraction of features from GunPoint dataset using null convolution.

**Figure 3:** The general flow of the algorithm.

**Figure 4:** Experimental results of two multimodal English feature structures using different fusion methods.

**Figure 5:** Comparative experimental results of four fusion methods using multimodal.

**Figure 6:** Statistics of grade means. (a) Pretest English score; (b) posttest English score.

**Figure 7:** Results of the test for differences in grade means.

**Figure 8:** Experimental results. (a) Experimental class; (b) control class.

**Figure 9:** Performance evaluation of the algorithm in this article compared with other algorithms.

**Table 1:** Structural hyperparameters of multimodal neural network LSTM-FCN.

LSTM module		FCN module		
Level	Number of neurons	Level	Convolution kernel size	Number of convolution kernels
1	32	1	10 *∗* 2	256
2	64	2	8 *∗* 1	128
3	128	3	5 *∗* 2	256

**Table 2:** Evaluation of instructional design activities.

Serial number	Evaluation type	Teaching link	Teacher evaluation dimension	Student evaluation
1	Notice	English preteaching activities	Does it attract attention?	Attention intensity
2	Association	English teaching content presentation stage	Is the content of English teaching relevant to learning?	English teaching content is consistent with learning
3	Self-confidence	English learner engagement stage	Are our teaching activities targeted?	Improve self-confidence in using English
4	Satisfaction	English evaluation and follow-up activities	Is the teaching evaluation reasonable?	English learning satisfaction

## Data Availability

The data used to support the findings of this study are available from the corresponding author upon request.
